The article "The Analysis of the Influence of Odorant’s Complexity on Fractal Dynamics of Human Respiration" was retracted in 2018. Reason: lack of ethics approval or compliance.

# The Analysis of the Influence of Odorant’s Complexity on Fractal Dynamics of Human Respiration

**DOI:** 10.1038/srep26948

**Published:** 2016-05-31

**Authors:** Hamidreza Namazi, Amin Akrami, Vladimir V. Kulish

**Affiliations:** 1 School of Mechanical and Aerospace Engineering, Nanyang Technological University, Singapore; 2 School of Metallurgy and Material engineering, University of Tehran, Iran

## Abstract

One of the major challenges in olfaction research is to relate the structural features of the odorants to different features of olfactory system. However, no relationship has been yet discovered between the structure of the olfactory stimulus, and the structure of respiratory signal. This study reveals the plasticity of human respiratory signal in relation to ‘complex’ olfactory stimulus (odorant). We demonstrated that fractal temporal structure of respiration dynamics shifts towards the properties of the odorants used. The results show for the first time that more structurally complex a monomolecular odorant will result in less fractal respiratory signal. On the other hand, odorant with higher entropy will result the respiratory signal with lower entropy. The capability observed in this research can be further investigated and applied for treatment of patients with different respiratory diseases.

One useful approach to study the scaling properties of many biological time series is to apply methods derived from the concept of self-similar (fractal) processes^1^,^2^,^3^,^4^,^5^. The fractal behavior shows the long-range correlations in these time series, which means the fluctuations in time series would be correlated with variations of hundreds of point earlier (presence of memory), and the correlations strength would decay in a power law manner.

The respiratory time series as the feature of respiratory system is governed as the result of inhalation and exhalation. The measurements of respiration time series (inter breath interval) reveal a combination of randomness and order, characteristic of fractal random processes^6^,^7^. For instance, Szeto *et al*. found out that breathing data on fetal lambs is fractal^8^. In another research, West *et al*. investigated that the fractal dimension of inter-breath intervals (IBI) and R–R intervals (RRI) decreases with increasing levels of exercise and is unaffected by hyperbaric exposure^9^. In case of analysing the effect of age and gender, Peng *et al*. found out that IBI time series in case of healthy elderly male has smaller value of fractal dimension compared to the young male, young female, and elderly female subjects^10^. Analysing the fractal properties of breathing data during sleep by Larsen *et al*. showed that fractal properties of IBI time series do not differ with sleep state for infants. Based on the observations they suggested that some of the respiratory variability that occurs during sleep in infants may be the product of deterministic processes^11^. See also^12^,^13^. In general, respiration time series like most physiological processes has a fractal dimension between D = 1 (regular process) and D = 1.5 (an uncorrelated random process).

The article "The Analysis of the Influence of Odorant’s Complexity on Fractal Dynamics of Human Respiration" was retracted in 2018. Reason: lack of ethics approval or compliance.

On the other hand, some researchers have focused on analysing the entropy of respiration time series. Caldirola *et al*. found out patients with panic disorder show greater entropy in baseline respiratory patterns, which reflects higher levels of irregularity and complexity in their respiratory function^14^. In another study, Angelini *et al*. showed that multi scale entropy calculated on lung volume time series significantly differs in patients and healthy subjects, and confirmed the complexity-loss theory of aging and disease^15^. In analysing the relative contributions of maturation to the dynamic behaviour of respiration during ontogeny, Akay *et al*. found out that the entropy were high during the first seven days of the postnatal age, and decreased for the 12–19 days, and increased during subsequent 26–31 days age. They suggested the unique decrease in the entropy values in 12–19 days age could be due to a reduction in the number of dendritic terminals per cell for this age range^16^. By computing the approximate entropy, Burioka *et al*. showed that respiratory movements are more regular during stage IV sleep than during other stages of consciousness^17^. See also^18^,^19^.

Besides all efforts done on analysis of breathing time series, no work has been done relating the complexity of stimuli (odorant in this research) to the complexity of respiratory time series. In this research we hypothesize that complexity of odorant should affect the breathing complexity. To test this hypothesis, we examine the quantitative relationship between the structural complexity of odorants and the fractal nature of respiratory signals. In the second step of this research we chose entropy as a tool in order to link the entropy of odorant with the entropy of respiratory signal.

## Method

In this research in order to analyse the influence of different odorants’ complexities on fractal dynamics of human respiration we need to quantify the odorant’s complexity. We do this job by considering the molecular complexity as an index of how complicated an odorant molecular structure is. This complexity is based on bond connectivity, diversity of non-hydrogen atoms and symmetry. In general, molecules and compounds that are small and/or highly symmetric with few distinct atom types (or elements) have low complexity. Here, we use Bertz formula for calculation of odorant molecular complexity^20^:



In equation (1), *C* is molecular complexity, *C*_*n*_ stands for skeletal complexity which is a function of bond connectivity (*n*) and *C*_*e*_ is a function of element diversity or kinds of atoms. *C*_*n*_ and *C*_*e*_ are composed of two terms which are an overall complexity term and a symmetry term subtracted from it, so as to reduce skeletal complexity (*C*_*n*_) or element diversity (*C*_*e*_) when the molecule is symmetric or atoms of the same kind are present.

The article "The Analysis of the Influence of Odorant’s Complexity on Fractal Dynamics of Human Respiration" was retracted in 2018. Reason: lack of ethics approval or compliance.

Another property that we consider about odorant is entropy. Based on third law of thermodynamic, at absolute zero, 0 °K, all substances are assumed to have zero entropy since at that temperature mobility of electrons, atoms or molecules of a compound is zero. So, whatever factor (such as temperature) tended to increase mobility of electrons, atoms or molecules of a compound causes to increase entropy of that compound. For instance, when a substance is warmed from, 0 °K, more kinetic energy is added to its electrons, atoms and molecules, so its entropy increases alongside its temperature.

Here we have two features for investigation about odorants which are molecular complexity and entropy. In order to analyse the influence of odorants we use these two features versus fractal dimension and entropy for respiratory signals.

In this research we do our analysis on inter breath interval (IBI) time series. This time series maps the time period for one complete cycle of respiration (end-to-end inspiration) versus time or interval number. The algorithms for generation and analysis of IBI time series are described in data analysis section.

### Data collection

Subjects in this research consisted of 20 women and 20 men (age 25 ± 1 years) with general health condition. The subjects were non-smoker and free of any known neurological, cardiovascular (checked through ECG) and respiratory diseases and didn’t drink alcohol or caffeine-containing beverages for more than 48 hours before the recording session.

All procedures were approved by the Internal Review Board of Nanyang Technological University and the approval for experimentation involving human subjects was issued by the university. The study was carried out in accordance with the approved guidelines. The nature of study was explained to participants before the experiments and then the written informed consent was obtained from them. It is noteworthy that the identity of all subjects remains confidential.

In this research we choose five odorants. Then, on one side we study the variations of odorants’ complexity versus IBI time series fractal dimension. On the other side, we study the variations of odorants’ entropies versus IBI time series approximate entropy.

The article "The Analysis of the Influence of Odorant’s Complexity on Fractal Dynamics of Human Respiration" was retracted in 2018. Reason: lack of ethics approval or compliance.

All experiments were done in an electrically shielded, acoustically isolated, and dimly illuminated room to insulate the subjects from all other external stimuli which may affect the respiratory signal. During the data collection subjects were sitting comfortably and instructed to focus on counting their respiratory rate and not allowed to talk or have any movement.

Since the vapor concentration of non-diluted odorants would be likely to correlate with molecular complexity, odorant concentrations were equalized by dilution in mineral oil according to their respective vapor pressure value, so as to achieve an approximate gas-phase partial pressure of 1 Pa. We presented each odorant in 10 ml vials and absorbed on scentless polypropylene fabric in order to optimize evaporation and air/oil partitioning. To further ensure that the resulting vapor concentrations did not differ according to molecular complexity, concentrations were measured for odorants using an olfactometer connected to a gas analyser. The output odorous air was fed into the gas analyser using a 4 mm tube (20 cm length). Each odorant was presented 5 times in the gas analyser with the duration of 3 sec and inter-stimulus interval of 2 min. No significant difference was observed in vapor concentration between odorants with different complexities.

In this research we used Respiratory Inductance Plethysmography (RIP) method for the collection of respiratory signals. RIP is an accurate plethysmography method which is frequently used to estimate lung volume from respiratory movements. In our experiments we used a RIP device (Respitrace, Ambulatory Monitoring, Ardsley, NY) which consists of a demodulator, an oscillator, and two wired elastic cloth bands. Signals were obtained from two elastic respiratory transducer bands, one placed around the rib cage under the armpits and the other around the abdomen at the level of the umbilicus (belly button). These transducers were connected to an oscillator and subsequent frequency demodulation device in order to obtain digital waveforms. In this research we used the summation of two governed signals (from two transducer bands). This summation was generated by sum channel of device. The recorded signal was sampled at 250 Hz and saved using the device software in the computer and used for analysis. The schematic of RIP method is shown in Fig. 1.

In the first round, the data collection was done without any stimulus. After that in order to test the effect of each odorant, we presented the odorant vial 1 cm below the subject’s nose and subjects sniffed at each vial presentation, and we collected the respiratory signal. We collected the data five times in case of each odorant with inter-stimulus interval of 2 min. After finishing the data collection for the first odorant we wait for 10 min and then we presented next odorant to subjects with the same procedure and continued to test all odorants. The data collections were repeated in the second day for each subject in order to examine the reproducibility of the results from experiments. By repeating the experiments in the second day totally 10 trials were collected in case of each odorant from each subject.

The article "The Analysis of the Influence of Odorant’s Complexity on Fractal Dynamics of Human Respiration" was retracted in 2018. Reason: lack of ethics approval or compliance.

### Data analysis

The respiratory signals are used as an indirect measurement of chest movement and lung volume. Since fluctuations of breath to breath cycle periods is of interest, it is necessary to map the respiratory signal only to relative changes in lung volume. So, from each digitized respiratory signal, the inter breath interval (IBI) was determined using an algorithm written in MATLAB (please see the supplementary material).

In fact, there are two issues which should be considered in analysis of respiratory time series. First, because of intrinsic respiratory oscillations as well as external fluctuations (due to environmental noise), the signals are very complex. Second, the signals are highly non-stationary. Figure 2 shows the digitized lung volume signal (time series) from a healthy subject.

In order to extract IBI time series, the developed algorithm should detect the main peaks of these non-stationary and noisy signals. In fact the detection of peaks is preferred, since the signal near its trough becomes relatively flat, and thus it is difficult to accurately identify the locations of the minimums. Thus, the algorithm should find all the local maxima which are correspond to the end points of inspiration.

However, due to signal noise and some transient physiologic interruptions there are some false peaks in the signal which algorithm should not consider them as local maxima. For instance, based on Fig. 2 in the expiration phase, while the respiratory signal moving downward, there may be brief increases of lung volume which creates local maxima in the signal. As it is clear in this figure, this local maxima is much smaller than the overall trend, so the program should not consider this local maxima and it should assume that the expiration phase persists. This behaviour can be seen also during the inspiration phase.

In the algorithm we adapt the moving average analysis technique that has been widely used in time series analysis^21^. This algorithm detects the main respiration peaks besides reducing noise in the signal. Considering a window of width *W* of the signal (*X*), the moving average over this window (*X*_*W*_) is defined as the average value of the signal at the preceding period of length *W*:



where *t* stands for the time.

The article "The Analysis of the Influence of Odorant’s Complexity on Fractal Dynamics of Human Respiration" was retracted in 2018. Reason: lack of ethics approval or compliance.

In order to detect the local peaks, two moving averages should be considered, one with a large window value *W*_1_ (slow-varying trend), and another one with a small window value *W*_2_ (fast-varying trend). For algorithm analysis, crossover points of these two moving averages are important. In fact, when the value of short-term moving average exceeds the value of long-term moving average, the signal is on an upward trend because the average of its recent history is greater than the average of its longer-term history. The values of short-term moving average diverge more and more as the signal continue on its upward behaviour. When the value of short-term moving average has the maximum difference with the value of long-term moving average, the signal is around its peak. The two moving averages approach each other as the signal moves downward, and finally the value of long-term moving average exceeds the value of the short-term moving average. Each true respiration peak is located between the crossover points where the short term moving average crosses over to values above and then below the long-term moving average curve.

In fact, the locations of peak points of smoothed time series generated by subtracting two moving averages are same with the locations of original signal peaks.

It is noteworthy in order to smooth out the local maxima generated by noise and pauses, *W*_1_ and *W*_2_ should be chosen carefully. Also, in order to optimize our algorithm first we examined a small subset of data. Then, we applied the optimized window sizes to the complete database.

To correct some misdetection by the algorithm, we inspected the time series visually after the algorithm automatically found the main inspiratory peaks of the respiration cycles. After we removed the false peaks (it was less than 1%) from the signal, another program generates the IBI time series which shows the interval size (vertical axis) versus interval number (horizontal axis). It should be noted that subsequent analysis was not very sensitive to this small amount of missing data.

For further investigation we analyzed each subject’s IBI time series by another MATLAB based programs which compute fractal dimension and entropy of IBI time series based on Box counting method^22^ and approximate entropy techniques^23^ respectively which are widely used in analysis of fractal time series (please see the supplementary material).

The article "The Analysis of the Influence of Odorant’s Complexity on Fractal Dynamics of Human Respiration" was retracted in 2018. Reason: lack of ethics approval or compliance.

### Statistical Analysis

Mean values for the dependent variables (fractal dimension and approximate entropy of IBI time series) were compared across no odorant and odorant breathing conditions with a one-way fixed-effect ANOVA. Mauchly’s test (*α* = 0.05) was conducted in order to test for sphericity. Trend analysis was performed across conditions when ordered according to the properties of the olfactory stimuli. For a repeated measures design, we used Omega squared (*ω*^2^) as an unbiased measure of effect size suitable for small samples; In order to do pairwise comparisons effect size, *r*, was used. All statistical analyses were performed using SPSS software.

## Results

In this research in order to analyze the effect of odorant’s molecular complexity and entropy on respiratory signal fractal dimension and entropy respectively, five pleasant odorants (Fig. 3) have been selected from Fenaroli’s Handbook of Flavor Ingredients^24^, which is a reliable and standard reference. The book includes expanded information on aroma and taste thresholds, and the most current regulatory information. Three dimensional molecular drawings were obtained from PubChem database Table 1 displays molecular complexity and entropy of the selected odorants.

As can be seen in Table 1, molecular complexity of selected odorants varies between 19.9 (Amyl alcohol) and 135 (Diethyl succinate). Molecular complexity values in this study were computed based on James B. Hendrickson *et al*. work^25^. As was mentioned before (also look at Fig. 3), in general, molecules and compounds that are small and/or highly symmetric with few distinct atom types (or elements) have low complexity. For instance, at the molecular level, Diethyl succinate (C8H14O4) is more complex than Amyl alcohol (C5H12O) because it is heavier and less symmetric than Amyl alcohol.

Also, as can be seen in Table 1, the entropy of selected odorants varies between 85.55 (Benzyl alcohol) to 136.29 (Diethyl succinate). In this study, the value of each odorant’s entropy in 25 °C was governed from (http://realtime.molinstincts.com/). As it is clear in Table 1, there is not any coupling between complexity and entropy variations of odorants.

No difference was observed between male and female subjects. Mauchly’s test indicated that the assumption of sphericity had not been violated for either outcome variable (fractal dimension & approximate entropy). Figure 4 shows the variation of mean of IBI time series fractal dimension in case of different odorants (on the left side), and the molecular complexity of odorants (on the right side). The results indicate the mean of all data governed from subjects in case of each odorant.

The article "The Analysis of the Influence of Odorant’s Complexity on Fractal Dynamics of Human Respiration" was retracted in 2018. Reason: lack of ethics approval or compliance.

Considering *F*_*crit*_(5,234) = 2.25 at *α* = 0.05, based on Table 2 the result of statistical analysis [*F*(5,234) = 82.5, p = 0.001] indicates that there was a significant effect of olfactory stimulus on the fractal exponent of IBI time series, with an effect size *ω*^2^ = 0.57.

As it is clear in Fig. 4, in general, breathing an odorant decreases the IBI fractal dimension. A significant linear trend between smelling conditions was observed (p = 0.003), indicating that Diethyl succinate smelling condition yielded lower fractal dimension of IBI time series than Dimethyl succinate smelling condition, followed by Butyl lactate, Benzyl alcohol and Amyl alcohol smelling conditions respectively. Effect size calculations between conditions suggest that Diethyl succinate breathing condition led to greatest changes in the IBI time series fractal exponent, observed across all Diethyl succinate comparisons (Table 3). In overall, the IBI time series fractal dimension decreases more by choosing odorants with higher molecular complexity. As fractal dimension stands for the complexity of a system, so it can be said that complexity of respiratory signal decreases more by choosing odorants with higher molecular complexity.

In another comparison, Fig. 5 shows the variations of IBI time series approximate entropy in case of different odorants (on the left side), and the odorants’ entropy (on the right side).

Considering *F*_*crit*_(5,234) = 2.25 at *α* = 0.05, based on Table 4 the result of statistical analysis [*F*(5,234)=95, p = 0.001] indicates that there was a significant effect of olfactory stimulus on the approximate entropy of IBI time series, with an effect size *ω*^2^ = 0.44.

As it is clear in Fig. 5, in general, breathing an odorant decreases the IBI time series approximate entropy. A significant linear trend between smelling conditions was observed (p = 0.0001), indicating that Diethyl succinate smelling condition yielded lower approximate entropy of IBI time series than Butyl lactate smelling condition, followed by Dimethyl succinate, Amyl alcohol and Benzyl alcohol smelling conditions respectively. Effect size calculations between conditions suggest that Diethyl succinate breathing condition led to greatest changes in the IBI time series entropy, observed across all Diethyl succinate comparisons (Table 5). In overall, the IBI time series approximate entropy decreases more by choosing odorants with higher entropy.

In summary, an adaptation occurred in respiration dynamics as a result of olfactory stimulation, where the odorants with higher molecular complexity/higher entropy will have greater influence on the complexity and entropy of human respiration respectively.

The article "The Analysis of the Influence of Odorant’s Complexity on Fractal Dynamics of Human Respiration" was retracted in 2018. Reason: lack of ethics approval or compliance.

## Discussion

In this research for the first time we analyzed the influence of odorant’s molecular complexity on the complexity of respiration time series. We did this job by analysing the odorant’s molecular complexity and IBI time series fractal dimension. The result of our analysis showed that by choosing an odorant with higher molecular complexity, the respiration signal is less complex, having smaller value of fractal dimension. On the other hand, we also investigated the behaviour of variations of respiration time series approximate entropy versus odorant’s entropy. The similar trend was observed in this case also, where by choosing an odorant with higher entropy, the entropy of respiration time series will decrease more. Statistical analysis also showed that odorant with higher molecular complexity or higher entropy has greater effect on fractal dynamics and entropy of respiratory signal respectively. In overall it can be said that there is a coupling between odorant’s complexity and IBI time series fractal dimension. Also, there is a coupling between odorant’s entropy and IBI time series approximate entropy.

The reason behind what was observed in this research can be investigated by linking to the nervous system. In fact when we smell an odorant, it is sensed by a patch of olfactory receptor neurons at the top of nasal passage behind nose. These neurons are out in the open where they can come into contact with the air. They have hair-like projections called cilia that increase their surface area^26^. An odorant molecule binds to these cilia to trigger the neuron and then a message will be sent to the brain in the form of a signal and causes we perceive a smell. In^3^ we showed that when human senses an external stimulus the value of the Hurst exponent for the EEG signal increases from 0.5. By increasing the Hurst exponent the fractal dimension decreases. We believe that when human smells an odorant with higher molecular complexity or higher entropy, this stimulus will have stronger effect on human brain, so accordingly the EEG signal will have smaller value of fractal dimension or entropy respectively. Thus, these stronger effects on human brain will accordingly stimulate the human lung more. So, the human respiration signal which is governed from lung volume variations will have smaller value of fractal dimension or entropy respectively. This hypothesis needs to be worked on more by simultaneous analysis of the effects of different odorants with different complexities on human EEG and respiratory signals.

Here we did our analysis in case of healthy subjects. These experiments can be further applied in case of subjects with some respiration diseases in order to investigate how much the odorant’s complexity or entropy affects the respiration system. Also, these analyses would guide on-going efforts to develop realistic models of respiratory control. In general, increased understanding of the relationship between odorants and the respiratory system shall speed up clinical practice in drug and design development which yields to therapy of different respiration diseases.

The article "The Analysis of the Influence of Odorant’s Complexity on Fractal Dynamics of Human Respiration" was retracted in 2018. Reason: lack of ethics approval or compliance.

## Additional Information

**How to cite this article**: Namazi, H. *et al*. The Analysis of the Influence of Odorant’s Complexity on Fractal Dynamics of Human Respiration. *Sci. Rep*. **6**, 26948; doi: 10.1038/srep26948 (2016).

## Supplementary Material

Supplementary Information

Supplementary Dataset 1

Supplementary Dataset 2

Supplementary Dataset 3

Supplementary Dataset 4

Supplementary Dataset 5

Supplementary Dataset 6

## Figures and Tables

**Figure 1:** Schematic of RIP method.

**Figure 2:** The digitized respiratory signal.

**Figure 3:** Molecular structure of selected odorants.

**Figure 4:** IBI time series fractal dimension in case of different odorants (on the left side), and the molecular complexity of odorants (on the right side). Error bars are standard deviations.

**Figure 5:** IBI time series approximate entropy in case of different odorants (on the left side), and the odorants’ entropy (on the right side). Error bars are standard deviations.

**Table 1:** Molecular complexity and entropy of selected odorants.

Name	Compound	Molecular complexity	Entropy
Amyl alcohol	C5H12O	19.9	95.38
Benzyl alcohol	C7H8O	55.4	85.55
Butyl lactate	C7H14O3	101	125.86
Dimethyl succinate	C6H10O4	114	118.24
Diethyl succinate	C8H14O4	135	136.29

**Table 2:** The result of ANOVA test in case of IBI time series fractal dimension (95% confidence interval).

	SS	df	MS	F	p
Between	0.824	5	0.165	82.5	0.001
Within	0.579	234	0.002		
Total	1.403	239			

**Table 3:** Effect sizes for pairwise comparisons in analysis of IBI time series fractal dimension.

Condition	Effect size (r)
No odorant vs. Amyl alcohol	0.58
No odorant vs. Benzyl alcohol	0.60
No odorant vs. Butyl lactate	0.82
No odorant vs. Dimethyl succinate	0.83
No odorant vs. Diethyl succinate	0.90
Amyl alcohol vs. Benzyl alcohol	0.10
Amyl alcohol vs. Butyl lactate	0.56
Amyl alcohol vs. Dimethyl succinate	0.60
Amyl alcohol vs. Diethyl succinate	0.75
Benzyl alcohol vs. Butyl lactate	0.43
Benzyl alcohol vs. Dimethyl succinate	0.58
Benzyl alcohol vs. Diethyl succinate	0.67
Butyl lactate vs. Dimethyl succinate	0.22
Butyl lactate vs. Diethyl succinate	0.51
Dimethyl succinate vs. Diethyl succinate	0.23

**Table 4:** The result of ANOVA test in case of IBI time series approximate entropy (95% confidence interval).

	SS	df	MS	F	p
Between	0.475	5	0.095	95	0.001
Within	0.326	234	0.001		
Total	0.801	239			

The article "The Analysis of the Influence of Odorant’s Complexity on Fractal Dynamics of Human Respiration" was retracted in 2018. Reason: lack of ethics approval or compliance.

**Table 5:** Effect sizes for pairwise comparisons in analysis of IBI time series approximate entropy.

Condition	Effect size (r)
No odorant vs. Benzyl alcohol	0.29
No odorant vs. Amyl alcohol	0.62
No odorant vs. Dimethyl succinate	0.76
No odorant vs. Butyl lactate	0.94
No odorant vs. Diethyl succinate	0.95
Benzyl alcohol vs. Amyl alcohol	0.25
Benzyl alcohol vs. Dimethyl succinate	0.52
Benzyl alcohol vs. Butyl lactate	0.70
Benzyl alcohol vs. Diethyl succinate	0.76
Amyl alcohol vs. Dimethyl succinate	0.40
Amyl alcohol vs. Butyl lactate	0.66
Amyl alcohol vs. Diethyl succinate	0.74
Dimethyl succinate vs. Butyl lactate	0.19
Dimethyl succinate vs. Diethyl succinate	0.40
Butyl lactate vs. Diethyl succinate	0.41
